This article has been retracted.

# HBsAg Inhibits the Translocation of JTB into Mitochondria in HepG2 Cells and Potentially Plays a Role in HCC Progression

**DOI:** 10.1371/journal.pone.0036914

**Published:** 2012-05-15

**Authors:** Yun-Peng Liu, Xiao-Ning Yang, Amarsanaa Jazag, Jin-Shui Pan, Tian-Hui Hu, Jing-Jing Liu, Bayasi Guleng, Jian-Lin Ren

**Affiliations:** 1 Department of Gastroenterology, Zhongshan Hospital affiliated to Xiamen University, Xiamen, Fujian Province, China; 2 Medical College of Xiamen University, Xiamen, Fujian Province, China; 3 National Institute of Medical Research, 3rd General Hospital, Ulaanbaatar, Mongolia; Aix-Marseille University, France

## Abstract

**Background and Aims:**

The expression of the jumping translocation breakpoint (JTB) gene is upregulated in malignant liver tissues; however, JTB is associated with unbalanced translocations in many other types of cancer that suppress JTB expression. No comprehensive analysis on its function in human hepatocellular carcinoma (HCC) has been performed to date. We aimed to define the biological consequences for interaction between JTB and HBsAg in HCC cell lines.

**Methods:**

We employed the stable transfection to establish small HBsAg expressing HepG2 cell line, and stably silenced the JTB expression using short hairpin RNA in HepG2 cell line. The effects of JTB and small HBsAg in vitro were determined by assessing cell apoptosis and motility.

**Results:**

Silencing of JTB expression promoted cancer cell motility and reduced cell apoptosis, which was significantly enhanced by HBs expression. Expression of HBsAg inhibited the translocation of JTB to the mitochondria. Furthermore, silencing of the JTB resulted in an increase in the phosphorylation of p65 in HepG2 cells and HepG2-HBs cells, whereas HBsAg expression decreased the phosphorylation of p65. The silencing of JTB in HepG2-HBs cells conferred increased advantages in cell motility and anti-apoptosis.

**Conclusion:**

HBsAg inhibited the translocation of JTB to the mitochondria and decreased the phosphorylation of p65 through the interaction with JTB, After JTB knockdown, HBsAg exhibited a stronger potential to promote tumor progression. Our data suggested that JTB act as a tumor suppressor gene in regards to HBV infection and its activation might be applied as a therapeutic strategy for in control of HBV related HCC development.

## Introduction

Complications of chronic HBV (CHB), including liver failure and hepatocellular carcinoma (HCC), which is one of the greatest risk factors for the development of HCC and the 10^th^ leading cause of mortality worldwide [1], [2], [3]. In the past two decades, a number of strong findings have shown that the X protein (HBX) acts as a transactivation factor and is clearly associated with tumorigenesis [4], [5], [6]. Functions in the carcinogenesis of other proteins, such as HBs, that are encoded by HBV are also related to liver tumor development [7], [8], [9], [10], [11]. HBV encodes three envelope proteins in the pre-S/S open reading frame, which are named the large, middle, and small surface proteins [7]. A number of truncated surface gene mutants with a partially deleted pre-S region have been identified; one of the major mutant types is the deletion of the pre-S2 region (pre-S2D). These pre-S2D mutants have become increasingly prevalent in the serum and liver tissues of patients with chronic HBV infection and HCC [12], [13]. The overexpression of pre-S2D (S2 characterized by the deletion of the pre-S2 region) large surface proteins has been demonstrated in the induction of endoplasmic reticulum (ER) stress [14], oxidative stress, DNA damage [15], COX-2 expression [16], cyclin A expression [17] and the degradation of p27Kip1 [18]. These results suggest that the expression of the HBV large surface protein, especially the pre-S2D mutant, might be important for hepatocarcinogenesis. However, determining putative additional roles for the S protein require further investigation.

Current cytogenetic evidence indicates the important role of the 1q21-q22 region in drug resistance [19], tumor metastasis [20] and a shorter duration of patient survival. Therefore, the function of the genes that are located proximal to this region may be associated with the process that accounts for the frequent translocation of the region in many types of tumors. A comparative genomic hybridization analysis of HCC indicates frequent gains of 1 q and an amplicon at 1q21-q22 [20]. Jumping translocation breakpoint (JTB) is a gene that is located on human chromosome 1 at q21 and undergoes an unbalanced translocation. Although JTB expression is suppressed in many cancers of different organs [21], [22], some studies have reported the overexpression of JTB in cases of hepatocellular carcinoma [20]. Therefore, the biological function of JTB remains unclear. Previous studies have raised the possibility that aberrations in the structure or expression of JTB induce neoplastic changes in cells, such as deregulated cell growth and/or death through mitochondrial dysfunction [22].

Our previous studies have suggested that there is an interaction between HBsAg and JTB, such as a recombination event [23], and that JTB may play a critical role in oncogenesis in the liver. However, the role of the interaction between HBs and JTB in liver tumorigenesis remains unknown. In this study, we aimed to investigate the functional changes in HepG2 cells by evaluating the interaction between JTB and HBs.

## Materials and Methods

### Cell culture, treatment and transfection

HepG2, L-02, HuH-7 and GES cells were grown in DMEM medium, SGC7901 cell was in RPMI1640, and AGS cell was in F12K medium, respectively. All cells were cultured in mediums with 10% fetal calf serum at 37°C in a 5% CO_2_ humidified atmosphere. The HCC cell lines HepG2, L-02 and HuH-7 were provided by the Cell Bank of Shanghai Institute of Cell Biology, Chinese Academy of Sciences, Shanghai, China. The HCC cells were treated with 0.6 mM H2O2 for 8 h. The HepG2 cells were transfected with 2 μg of the pCMV-HBsAg vector using FuGENE HD (Roche, Indianapolis, IN) in six-well plates. After 48 hours of transfection, the cells were split 1∶10 and selected with 600 μg/mL G418 (Sigma, St Louis, MO) for 2 weeks. The G418-resistant colonies were pooled together, and the HBs-expressing clones were identified by immunoblotting and maintained with 600 μg/mL G418. HepG2 cells were transfected with siJTB (pcPUR+U6-siJTB) or a PU6 (pcPUR+U6-siRenilla) plasmid using the FuGENE HD (Roche, Indianapolis, IN). Puromycin (2.0 μg/ml) was used to screen stably transfected clones. The expression of the JTB protein was examined by Western blotting analysis using an antibody against JTB (these experiments were repeated three times) to validate the efficiency of the constructs to inhibit target gene expression.

### Stable knockdown of JTB

A plasmid containing an RNA interference sequence that targeted HepG2 was constructed as previously described [24], [25], and a line of stable HepG2 knockdown cells were also established as previously described [26], [27]. One pair of the siJTB sequence was Forward primer, 5′- CACCGCGGAAGAGTGTTCTTCATA CGTGTGCTGTCCGTATGGAGAGCACTCTTCTGCTTTTT -3′, and Reverse primer, 5′- GCATAAAAAGCAGAAGAGTGC TCTCCATACGGACAGC ACACGTATGAAGAACACTCTTCCGC -3′. HepG2 cells were transfected with pcPUR+U6-siJTB or pcPUR+U6-siRenilla (control) and selected as puromycin-resistant pools. Quantitative reverse transcription-PCR (qRT-PCR) was performed to confirm the JTB mRNA suppression using the primers 5′- CGGGCTAAAACTACCCCTGAG -3′ and 5′-TGAGCGGCAGCTTTTGAACT-3′.

### Western blot analysis and co-immunoprecipitation

Cells were re-suspended in lysis buffer containing a protease inhibitor cocktail, and the extracted proteins were separated using 10–15% SDS–PAGE gels. β-actin was used as a loading control. Antibodies against β-actin, tubulin, coxIV, bcl-XL, caspase-9, cytoC, MMP-2, PARP, p-p65 (ser536) and p65 were obtained from Cell Signaling Technology; JTB antibody was obtained from Sigma Aldrich. Co-immunoprecipitation was performed using whole-cell lysates and antibodies against JTB and HBsAg. The immunoprecipitation was performed with A/G agarose beads that were coated with anti-JTB or anti-HBs, and the proteins were detected using anti-JTB and anti-HBs antibodies via western blot analysis. Mouse or rabbit immunoglobulin IgGs were used as negative controls.

### Flow cytometric and apoptosis assays

HCC cells were used for the apoptosis assays. The HCC cells were seeded into a 24-well culture dish and treated with 0.6 mM H_2_O_2_ for 8 h. The treated cells were washed with PBS three times followed by trypsinization. The harvested cells were stained with the Annexin V-FITC apoptosis assay kit (Kaiji Corp., Nanjing, China) according to the manufacturers' manual. Finally, the cells were assessed for apoptosis ratios using flow cytometry. The experiments were performed in triplicate.

### RNA extraction, reverse transcription and real-time PCR

Briefly, first-strand cDNA was synthesized using the ImProm-II reverse transcription system (Promega, Madison, WI) and was subjected to quantitative PCR using a Light Cycler 480 system (Roche, Indianapolis, IN). The primer sequences were as follows: MMP-2, forward 5′-TGATCTTGACCAGAATACCATCGA- 3′ and reverse 5′-GGCTTGCGAGG GAA G AAGTT- 3′; GAPDH: forward 5′-CAAGGTCATCCATG ACAACTTTG- 3′ and reverse 5′-GTC CACCACCCTGTTGCTGTAG-3′. Bcl-XL: forward 5′- GTGAATGGAGCCACTGCGC A- 3′ and reverse 5′-CCCCATCCCGGAAGAGTTCA- 3′.

### Transwell invasion and wound healing

Transwell invasion assays were performed with 8.0-μm pore inserts in a 24-well transwell plate. For this assay, the HCC cell lines were added to the upper chamber of a Transwell with 0.5 mg/mL collagen type l (BD Bioscience, San Jose, CA)-coated filters for the invasion assay. DMEM with 10% fetal bovine serum and 1% of each antibiotic was added to the lower chamber, and the cells were allowed to incubate for 16 hours. Invading cells were quantified after Gentian violet staining. Each experiment was performed in triplicate, and the data were expressed as mean values. A wound-healing assay was performed in 24-well plates. Tumor cells in medium containing 10% FBS were seeded into 24-well plates (Corning, CA). After the cells grew to confluence, made the wounds using sterile pipette tips, then, cells were washed with PBS and refreshed with medium with 10% FBS. The photographs were token at 0 and 24 h.

### Isolation of cytosolic and mitochondrial fractions

The isolation of cytosolic and mitochondrial fractions was performed using the ApoAlert kit. After H_2_O_2_ treatment, the cells were plated in 75-cm^2^ flasks and harvested by trypsinization. A total of 5×10^7^ cells were centrifuged at 600× g for 5 min at 4°C. The pellet was resuspended in 0.8 ml of ice-cold fractionation BufferMix, incubated on ice for 15 min, and homogenized with a Dounce tissue grinder on ice. The homogenate was subsequently transferred to a microcentrifuge tube and centrifuged at 700× g for 10 min at 4°C. The supernatant was collected and transferred to a fresh microcentrifuge tube and centrifuged at 10,000× g for 25 min at 4°C. The cytosolic fraction was collected, and the pellet, representing the mitochondria-containing fraction, was resuspended in 100 μL of fractionation BufferMix. The protein concentration was determined using the BCA method with bovine serum albumin as standard. The cytochrome c in the cytosolic and mitochondrial fractions was analyzed using western blot analysis.

### Cell immunofluorescence analysis

For cell immunofluorescence, 5×10^4^ HepG2 and HepG2-HBs cells were plated onto coverslips in 24-well plates for 24 hours. The cells were fixed in 4% paraformaldehyde for 10 minutes, permeabilized with 0.1% Triton X-100 for 10 minutes, and blocked with 10% BSA for 30 minutes. Next, the cells were incubated at room temperature with or without primary anti-JTB, anti-HBs or anti-coxIV antibodies for 1 hour followed by the respective secondary antibodies Texas Red goat anti-mouse antibodies and fluorescein isothiocyanate (FITC). The nuclei were counterstained with DAPI dye before the slides were mounted with the FluorSave reagent. The slides were observed under an Olympus FV-500 fluorescent microscope.

### Luciferase reporter gene assays

The transcriptional activity of the p65-responsive element was assessed using the p65 reporter assay. Briefly, the p65 and negative control reporter plasmids were separately transfected into HCC cells in replicate wells using Lipofectamine 2000 reagent (Invitrogen). Two days after transfection, the luciferase activity was determined using the dual-luciferase reporter assay system (Promega).

### Statistical analysis

The data were expressed as the mean ± standard error of the mean (SEM). Experimental differences were analyzed using SPSS v11 with the 2-tailed t-test and with *P*<0.05 defined as the selected level of significance.

## Results

### JTB binds HBs, and HBs expression reduces the mitochondrial localization of JTB

To explore the expression of JTB in different liver cancer cell lines, we examined the nomal liver cells and several liver cancer cell lines on JTB expression by western blotting. Meanwhile we established HepG2 stable cell line expressing HBsAg and silenced JTB expression using short hairpin RNA stable produced in HepG2 cell line. The JTB expression in the HCC cell lines recapitulated the pattern of expression in the human HCCs. The cell lines expressed high (HepG2 and Huh7 cells), intermediate (L-02 cells), or low-to-undetectable (HepG2-JTBi and HepG2-HBs-JTBi cells) levels of JTB. In addition, gastric cancer SGC7901 and AGS cell lines showed the lower expression level of JTB compared with normal gastric GES cell (Figure 1 A).

We have previously shown that the JTB protein binds to the HBV surface antigen (HBsAg). However, we used JTB delivered exogenously by transfection. To further illustrate the relationship between the combination of JTB and HBsAg. Recently, we used the endogenous JTB in HepG2 cells to detect whether a combined effect of the endogenous JTB protein and HBs existed. The cell lysates were subjected to immunoprecipitation with the anti-JTB antibody followed by western blot analysis with anti-JTB and anti-HBs antibodies; another set of cell lysates were also subjected to immunoprecipitation with the anti-HBs antibody followed by western blot analysis with anti-JTB and anti-HBs antibodies. The whole-cell lysate was used as a positive control, and immunoglobulin IgG was used as a negative control. The results showed that the anti-JTB antibody precipitated HBs and that the anti-HBs antibody precipitated JTB (Figure 1B).

**Figure 1:** JTB interaction with HBs in HepG2 cells. (A) The expression levels of JTB in HCC cell lines and normal liver cell, JTB in gastric cancer cells and normal gastric cell were determined using western blot analysis. HBs was detected for stable transfected cells. β-actin was used as a loading control. (B) Immunoprecipitation was performed as described in the Materials and Methods section. JTB and HBs were detected by western blot analysis. The whole-cell lysate was used as a positive control. (C) A western blot showing the distribution of JTB in the cytosolic and mitochondrial subfractions. Tubulin and coxIV were used as cytosolic and mitochondrial markers, respectively. (D) The effects of JTB on the mitochondrial localization and co-localization of JTB and HBs. Cellular localization by the immunocytochemical analysis of JTB and HBs in HepG2 cells using (a, b) FITC-labeled anti-JTB (green) and Texas red-labeled anti-coxIV (red) antibodies, (d, e) FITC-labeled anti-JTB (green) and Texas red-labeled anti-HBs (red) antibodies, (g, h) and FITC-labeled anti-JTB FITC (green) and Texas red-labeled anti-coxIV (red) antibodies under confocal microscopy. To label the nuclei, 4′,6-diamidino-2-phenylindole (DAPI) was used (blue). Bars, 10 μm.

Furthermore, we applied immunofluorescence confocal technology to prove the combination of HBsAg and JTB. We determined the localization of JTB in HBs-transfected HepG2 cells using western blot analysis (Figure 1C) and immunocytochemistry (Figure 1D). JTB was localized to the mitochondria (Figure 1D a, b and c), and HBs co-localized with JTB (Figure 1D d, e and f). The expression of HBs decreased the translocation of JTB to the mitochondria and caused the cytoplasmic accumulation of JTB, which inhibited the co-localization of JTB with the mitochondria marker cox IV (Figure 1D g, h and i). The change of JTB cellular localization could make effect on cell function. In the next experiments, we will explore the cell function involved apoptosis and motility after the change of cellular localization.

### JTB knockdown suppresses H_2_O_2_-induced apoptosis by increasing Bcl-XL

The exposure of cells to H_2_O_2_ induces apoptosis through pathways that involve the disruption of normal mitochondrial function. One key mechanism involves the opening of the mitochondrial permeability transition pores (PTPs) that allow the passage of some small pro-apoptotic molecules, such as cytochrome c into the cytoplasm [28], [29]. Previous studies have reported that the opening of PTPs increases when the mitochondrial membrane potential decreases [30].

To explore the role of JTB and interaction with HBsAg on cell apoptosis, we used H_2_O_2_ to induce oxidative stress which cause the cell apoptosis. The response to H_2_O_2_ -induced apoptosis in different liver cancer cell lines was examined by Flow cytometric and apoptosis assays. As shown in Figure 2A and B, the Annexin V signal significantly decreased in cells knocked down for JTB compared to cells transfected with the control pU6-sh plasmid. HBs expression enhanced the effect of decreasing the number of Annexin V-positive cells in the population of HepG2 cells. Our results show that JTB and HBs act cooperatively to reduce apoptosis. HBs expression was expected to reduce the sensitivity of a cell to H_2_O_2_-induced apoptosis after JTB knockdown, and HBs did not exhibit anti-apoptotic effects in the presence of JTB. Knockdown of JTB induced Bcl-XL upregulation(Figure 2C and D). Cytochrome c accumulated in the cytosol of vector-transfected cells and was markedly abundant compared to that found in the cytosol of cells knocked down for JTB (Figure 2E). In the cytoplasm, cytochrome *c* binds to APAF-1 to form an apoptosome, which activates caspase 9 (Figure 2F). H_2_O_2_-induced cell apoptosis was reduced in the cells with JTB knockdown, and the disruption of the mitochondrial transmembrane potential (MTP) and cytochrome c leakage were reduced. The anti-apoptotic gene Bcl-XL was also highly expressed. In the hepatoma cells, JTB expression protected the cells against H_2_O_2_ injury. This effect may be associated with the preservation of mitochondria. Upregulation of Bcl-XL plays a crucial confrontation to apoptosis. JTB regulate the Bcl-XL expression through some unknown pathway.

**Figure 2:** Stable knockdown of JTB in HCC cells decreases cell apoptosis. HepG2 cells were treated with 0.6 mM H_2_O_2_ for 8 h. (A) The percentage of apoptotic cells in HepG2 cells. (B) Quantification of apoptosis cells in different HepG2 cells. The percentage of apoptotic cells was determined using cyto-fluorimetric analysis with Annexin-V and PI labeling. The data were obtained from three analyses (*P<0.05). (C and D) The level of the Bcl-XL mRNA in HepG2 cells as measured using qRT-PCR. The results represent the mean of three amplifications and were calculated using the 2 exp^(−△△Ct)^ formula. β-actin mRNA in HepG2 cells was used as a control (*P<0.05). (E) Western blot analysis of the cytosolic and mitochondrial cytochrome c levels in HepG2 cells induced by H_2_O_2_ after 8h. (F) Uncleaved (p47) and activated caspase-9 (p37) were detected by western blot analysis in HepG2 cells induced by H_2_O_2_ after 8 h.

### Silencing of JTB increases cell motility, which is enhanced by HBs

To further explore the biological function of JTB, We determined the effects of HBs and JTB silencing on cell invasion and wound healing (Figure 3A–D). As expected, JTB silencing significantly promoted both of these processes, whereas HBs did not induce migration or invasion in HepG2 cells. To show the effect of JTB on HBs, we stably silenced JTB using its shRNA in the HepG2-HBs cells, which strongly express JTB. Invasion assays were performed to determine the effect of JTB silencing on cancer cell motility, and the cell numbers were counted (Figure 3C) and recorded (Figure 3A) using a microscope. As shown in Figure 3A and B, JTB knockdown increased cell migration and invasion, which was significantly enhanced by HBs expression. Furthermore, to explore the molecular mechanisms in cell migration and invasion, we examined whether JTB regulates cell motility through the MMP-2 protein and mRNA expression. We found that the level of MMP-2 expression was significantly enhanced in HBs+JTBi cells in comparison to pU6-JTBi cells (Figure 3E–F). These results suggest that JTB could regulate the expression of MMP2 and affect the cell motility, while the presence of HBsAg play has an important biological synergy function with JTB.

**Figure 3:** Transient knock-down of JTB promotes migration and invasion in the HCC cells expressing high levels of JTB. (A) Images and graphs (C, *P<0.05) from invasion assay at 16 h; (B) Images and graphs (D, *P<0.05) from migration assay the migrating ability of control cells at 24 h was considered as 1 in (D); The MMP-2 protein expression was detected using western blot analysis (E), and the mRNA expression was quantified using qRT-PCR (F).

### Silencing of JTB increases p65 activity, and HBs enhances this effection

Summarize the previous results, JTB and HBsAg have new biological functions on cell apoptosis and motility. We initially explore the possible associated signal transduction pathway. We examined the effect of JTB and HBs on NF-κB activation. Canonical NF-κB activation was assessed using phospho-immunoblot analysis (Figure 4A) and luciferase activity assay (Figure 4B). Immunoblot analysis for phospho-p65 revealed an increased phosphorylation of p65 in pU6-JTBi and HBs+JTBi cells, although the level of phospho-p65 was significantly increased in HBs+JTBi cells compared to that in pU6-JTBi cells. The same trends were demonstrated in luciferase activity assay. These results show the biological activity of HBs in HCC progression. The presence of JTB masked the function of HBs. In addition, we are trying to find more upstream signaling molecules. We used the protein chip technique to detect changes in the major protein kinase activities in different HCC cell lines, and the results of this experiment revealed that several protein kinases, such as AKT, ERK, RSK1, GSK-3β, showed dramatic changes in their level of phosphorylation (Figure 4C). Thus, we detected the phosphorylation level of three protein kinases using western blot analysis (Figure 4D), and the results were consistent with those obtained with the protein chip technique.

**Figure 4:** Activity of p65 and other protein kinases in HCC cell lines. The transcriptional activity of p65 was measured indirectly using luciferase reporter assays and normalized against TK-renilla. (A) Immunoblot analysis for phospho-p65 and total p65 protein expression. Increased phosphorylation of p65 was detected in both pU6-JTBi and HBs+JTBi cells, whereas HBs inhibited p65 phosphorylation. (B) Transcriptional activity of the p65 promoter in HepG2 cells using the luciferase activity assay was consistent with the level of p65 phosphorylation. The data were expressed as the mean of three experiments and as a percentage of the p65 promoter activity compared to that in the HepG2-vector cells (100%). (C) The results of the Human Phospho-MAPK Array Kit (R&D Systems, Inc.) In addition, we determined the relative levels of phosphorylated mitogen-activated protein kinases (MAPKs) and other serine/threonine kinases. (D) The phosphorylation levels of AKT, ERK and GSK-3β were detected by western blot analysis.

## Discussion

The hepatitis B surface antigen (HBsAg) was the Nobel Prize discovery that identified the hepatitis B virus (HBV) approximately 40 years ago. Currently, HBsAg remains the hallmark of overt HBV infection [3]. Hildt et al. found that the Pre-S2 members of the regulatory protein family, including L-HBs and truncated M-HBs, are transcriptional activators that trigger the activation of tumor promoters [31]. The small (S) protein is expressed at the highest levels and is predominant in virions and subviral particles. However, the role of S-HBs in HBV-induced oncogenesis is not well understood. Therefore, the present study was designed to verify the function of HBs via the interaction of HBs with JTB.

Our previous study had shown that the viral envelope protein HBs interacts with JTB. In addition, S-HBs and L-HBs functionally bind JTB, which presumably indicates that the binding site may be located in the S region of viral HBs [23]. JTB is upregulated in liver cancer cells [20], and previous research has demonstrated that JTB is downregulated in other cancer tissues [22]. It has been shown that the elevation of Sp1 protein expression is a critical factor in tumor development and growth and metastasis, and it is the promoter of JTB contains a sp1-binding site [21]. Therefore, JTB expression may be elevated in human tumors. In the current study, the overexpression of JTB reduced neoplastic changes in cells, such as regulated cell death via mitochondrial dysfunction. We also found that overexpression of JTB lead to apoptosis in normal liver L-02 cell line induced by H_2_O_2_, JTB can increase the activity of caspase9 and promote the cleavage of PARP (Figure S1 and data S1). When the JTB gene undergoes an unbalanced translocation, its expression is suppressed; therefore, we concluded that JTB is a tumor suppressor gene. The jumping translocation of the JTB gene eventually leads to the development of tumors to promote tumor differentiation and staging.

When we stably transfected the HepG2 cells with HBs, the JTB protein interacted with HBs and inhibited the translocation of JTB to the mitochondria. The interaction between JTB and its specific binding protein, HBs, mediates several cellular functions. Our data indicate the possibility that blocking JTB may increase the metastatic potential and reduce the apoptotic potential of cancer cells. However, transfection of HBs alone into HepG2 cells did not perturb apoptosis or metastasis. Surprisingly, blocking JTB in pCMV-HBs cells seems to enhance anti-apoptotic and metastastic activities compared to that in HepG2 cells. These results suggest that HBs has a biological activity that is JTB-independent. We showed that JTB inhibited the phosphorylation and reduced the biological activity of p65; thus, we speculate that the presence of HBs may sequester JTB in the cytoplasm and decrease the phosphorylation of p65. Blocking or knockdown of JTB may promote the HBs-mediated phosphorylation of p65.

NF-kB plays a well-known function in the regulation of immune responses and inflammation, but growing evidences support a major role in oncogenesis. In vitro, neutralizing the interaction of JTB and HBs significantly impaired the metastasis of liver cancer cells and cell apoptosis. This result suggests that JTB is important for the function of HBs in HCC cells and indicates the possibility that the strengthening of JTB/HBs interactions may be a strategy to prevent cancer cell metastasis and antiapoptosis. JTB expression reduces tumor metastasis and antiapoptosis by decreasing p65 activity. p65 regulates the expression of genes involved in many processes that play a key role in the development and progression of cancer such as proliferation, migration and apoptosis. The Bcl-XL protein plays an important role in maintaining the intergrity of mitochondrial thereby inhibiting the release of factors which activate the pro-apoptotic caspase cascade [32]. MMP-2 is known to play a crucial role in tumor invasion via its ability to degrade basement membrane collagens. It plays important roles in cancer development and aggression. p65 directly activates expression of the apoptosis inhibitor Bcl-XL [33] and matrix-modifying enzyme MMP-2 [34]. The activation of HBs following JTB knockdown may protect cell from apoptosis and trigger the degradation of extracellular matrix substrates.

To investigate the mechanism of regulation in p65 activity, we used protein chip technology to detect changes in signaling molecules that are associated with the MAPK pathways. We determined that HBs may phosphorylate AKT and ERK for activation. However, the pCMV-HBs cells were not protected from apoptosis and did not exhibit increased migration. We speculate that HBs activity was inhibited due to JTB. GSK-3 beta is phosphorylated in vitro at serine 9 by RSK1, resulting in its inhibition [35]. The activation of RSK1, which is involved in regulating cell survival and proliferation, lays at the end of the signaling cascade mediated by the extracellular signal-regulated kinase (ERK) subfamily of mitogen-activated protein (MAP) kinases [36]. HBs activated ERK signal pathways. But HBs may decrease p65 activity following the translocation of JTB into the cytoplasm. After JTB knockdown, HBs exhibited a stronger potential to promote tumor progression. We observed that there is a lower level of GSK-3βphosphorylation and higher level of p65 phosphorylation in HBs+JTBi cells. It has been reported that GSK-3β can phosphorylate the C-terminal domain (residues354–551) of p65 in vitro [37]. However, the role of the interaction between JTB and HBs in GSK-3βphosphorylation is unclear. This issue will be our research focus in the future. JTB protein and HBs play different roles in human HCC. HBs may act as an oncogene that is integrated into the human genome, whereas JTB is presumably a tumor suppressor gene. Therefore, therapeutic approaches that are aimed at eliminating HBs and/or reactivating JTB might be highly useful in the treatment of human liver cancer.

## Supporting Information

Figure S1 **Caspase9 activity and western blot analysis in L-02 cells induced by H_2_O_2_.**
(TIF)

Data S1 **Supplementary data.**
(DOC)
